# Application of Melatonin with N-Acetylcysteine Exceeds Traditional Treatment for Acetaminophen-Induced Hepatotoxicity

This article has been retracted.

**DOI:** 10.1155/2022/2791743

**Published:** 2022-09-02

**Authors:** Mengfei Chen, Jinfang Ke, Shilan Ma, Hua Chai, Liang Zhang, Ling Zhang

**Affiliations:** Department of Emergency, People's Hospital of Ningxia Hui Autonomous Region, Ningxia, China

## Abstract

Acetaminophen (APAP) overdose is one of the leading causes of acute liver damage. Given N-acetylcysteine (NAC) and melatonin (MLT) both have an attenuated value for APAP-induced liver toxification, where an optimized integrated treatment has not been well deciphered. Here, by giving a single dose of APAP (500 mg/kg) to wild-type male mice, combined with a single dose of 500 mg/kg NAC or 100 mg/kg MLT separately as the therapeutic method, this study aimed to investigate the effects of NAC and melatonin (MLT) alone or combined on acetaminophen (APAP)-induced liver injury. In this study, NAC and MLT both partially have an alleviated function in APAP-challenged liver injury. However, MLT's add-on role strengthens the hepatoprotective effect of NAC on APAP-induced liver damage and resolute the inflammatory infiltration. Meanwhile, the combination of two reagents attenuates the decreased glutathione (GSH) and activation of the p38/JNK pathway. The combination of MLT and NAC can further ameliorate APAP-induced liver injury, which provides a novel strategy for drug-induced liver injury (DILI).

## 1. Introduction

Various inflammatory mediators could aggravate liver damage during the process of APAP overdose intoxication [1]. In the clinical context, different conditions can lead to the impairment of liver function and the occurrence of acute liver injury. Drug poisoning is a leading cause of acute liver failure, where APAP overdose nearly accounts for 50% of all liver injuries [2].

Widely used in analgesics and antipyretics, APAP is considered effective in therapeutic doses [3], and the dose of APAP varying from 1 to 4 g/day is considered clinically safe [4]. Mainly metabolized by UDP-glucuronosyltransferase (UGT) and sulfotransferase (SULT), it can be expelled through urine [4]. However, APAP overdose can cause severe liver damage to both patients and laboratory animals [5]. As for the underlying mechanism behind hepatotoxicity, it is caused by the saturation of sulfation and glucuronidation metabolic pathways. More importantly, the production of N-acetyl-p-benzoquinone imine (NAPQI) during hepatotoxicity can be induced by some hepatic cytochrome P-450 (CYP) isoenzymes, especially CYP2E1 [6]. NAPQI depletes the GSH in a critical process and is regarded as an electrophile that binds covalently to essential proteins, which subsequently creates an environment conducive to oxidative stress that leads to hepatocyte death [5]. In particular, APAP causes mitochondrial ROS by affecting the ATP/ADP ratios and c-jun N-terminal kinase (JNK) activation, which can further aggravate liver damage [7, 8]. Excessive APAP intake not only causes metabolic acidosis but also elevated transaminases. In addition, it activates damage-related molecular patterns (DAMPs), produces various proinflammatory cytokines and chemokines, and consequentially amplifies liver damage [9].

At present, the following mechanisms are mainly identified as protective against APAP-induced liver damage: the stimulation of glutathione synthesis, CYP2E1 inhibition, HSP induction, and the inhibition of oxidative stress [10, 11]. The antioxidant N-acetylcysteine (NAC), a sort of cysteine prodrug, is clinically most used to treat APAP intoxication. Besides, it is also treated as what replenishes the intracellular stores of hepatic GSH [12]. The treatment should be administered intravenously in a timely manner and last 20 hours. Despite this, it can still lead to such adverse events as allergic reactions, nausea, vomiting, diarrhea or constipation, fever, headache, lethargy, and hypotension [13].

Melatonin (MLT) is responsible for various physiological processes and plenty of studies suggest the beneficial effects of melatonin on liver damage and diseases [14]. Shown as a free radical scavenger, MLT can produce antioxidant enzymes to become an antioxidant, including anti-lipid peroxidation and protein peroxidation [15]. Apart from that, MLT can also induce *γ*-glutamylcysteine synthetase (*γ*-GCS), the rate-limiting enzyme of GSH synthesis, thus increasing the concentration of cellular GSH in human vascular endothelial cells [16]. MLT treatment can significantly inhibit the APAP-induced activation of serine/threonine kinase receptor-interacting protein 1 (RIP1) and suppress JNK phosphorylation and mitochondrial Bax translocation, thus preventing AIF-dependent cell death [17].

As a leading cause of DILI, APAP overdose might result in acute liver failure and mortality. As an effective treatment for APAP-overdose patients, the administration of NAC is subject to some limitations in the protection against liver injury [6]. In this study, a new investigation was conducted based on a favorable combinator application of NAC with MLT in mitigating liver damage.

## 2. Methods

### 2.1. Animals and Liver Injury Model

Male wild-type C57BL/6 mice were purchased from Shanghai SLAC Laboratory, and mice liver injury models were constructed as previously reported [18]. APAP (obtained from Sigma-Aldrich) was dissolved in PBS at 55°C before the immediate heating to 37°C. Then, mice, after overnight fasting, received intraperitoneal (i.p.) PBS or APAP (500 mg/kg) injection. 500 mg/kg of NAC [9] (Sigma-Aldrich, i.p., 30 min before APAP injection) either separately or combined with 100 mg/kg of melatonin (MLT) [19] (Sigma-Aldrich, intragastrical, 30 min before APAP injection) was given to the required mice groups. These mice, after overnight fasting, only received i.g. PBS and were treated as a control group. All mice were sacrificed 24 hours or an indicated time after APAP injection by isoflurane inhalation (concentration of 5%) and cervical dislocation. No heartbeat was considered death in this study. The experiment was approved by the Laboratory Animal Ethical and Welfare Committee of Ningxia Medical University.

### 2.2. Liver Histology Analyses

Liver tissue was fixed in paraformaldehyde, and low to high concentration alcohol was used as a dehydrating agent to gradually remove water from tissue blocks. Then the tissue block was placed in the transparent agent xylene, which is soluble in alcohol and paraffin wax, to replace the alcohol in the tissue block with xylene, to dip wax embedding. Prepare a container (such as folding a small paper box), pour the melted paraffin into it, and quickly clip the paraffin-soaked tissue into it. After cooling, it solidifies into blocks. The embedded tissue blocks harden before they can be cut into very thin slices on a slicer. The embedded wax block is fixed on the slicer and cut into thin slices, usually 5–8 microns thick. HE staining is commonly used to increase the color difference of each part of tissue cell structure, which is convenient for observation.

### 2.3. Western Blot

Briefly, liver tissue was harvested and extracted by RIPA lysis buffer (Thermo Fisher). After protein BCA quantification (Thermo Fisher), the samples were separated by SDS-PAGE gel electrophoresis and immunoblotted to nitrocellulose membranes. Subsequently, the membranes obtained were blocked with 5% milk and incubated with 5% BSA dissolved antibodies overnight at 4°C. The antibodies used in this study are detailed as follows: *β*-actin, anti-Rabbit (all from Jackson, 1 : 10000), phosphor-p38 (CST,4511), p-38 (CST, 8690), phosphor-JNK1(CST, 9259), JNK1(CST, 3708), and RIP1(CST, 3708) (all from Cell Signaling Technology, 1 : 1000). Besides, the second antibodies were diluted in 5% BSA and incubated for 1 hour at room temperature.

### 2.4. Acute Toxicity Analyses and Inflammation Detection

Mice serum ALT, AST, and the activities of liver superoxide dismutase (SOD) and catalase (CAT) were detected using a biochemical kit (Nanjing Jiancheng Institute, China) in line with the applicable protocols. TNF*α* and IL-6 levels were tested using the ELISA kits provided by Neo Bioscience, China. In accordance with the commercially available protocol (ab118970, Abcam), malondialdehyde (MDA) was equivalently represented to indicate the lipid peroxide expression. The percentage of neutrophils was obtained through cytometrical flow. The flow antibodies CD11b and Ly6G were added as instructed and then detected by the machine. The populations were analyzed by using Cytoﬂex S Flow Cytometer (Beckman Coulter, USA), while the data was analyzed using a CytExpert software package.

### 2.5. Statistical Analysis

The data used in this study are all denoted as means ± SD through GraphPad Prism 9.0 (San Diego, USA). The one-way analysis of variance (ANOVA) and posthoc Tukey tests were conducted to analyze the difference between the two groups. When *p* values are less than 0.05, it would be treated as statically significant (^*∗*^means *p* < 0.05, ^*∗∗*^ means *p* < 0.01, ^*∗∗∗*^ means *p* < 0.001, respectively).

## 3. Results

### 3.1. MLT Strengthens the Hepatoprotective Effect of NAC in Liver Damage

Given MLT has been demonstrated as capable to interrupt APAP's toxicity [14], NAC is accepted as a standard method applied to treat acetaminophen-induced liver injury (AILI). Firstly, it was placed conditionally on the effect of combining MLT as the standard method with the mono treatment of NAC. In this study, APAP overdose could produce a satisfactory outcome of liver injury in wild-type (WT) mice, which exhibited a significantly elevated level of serum transaminase (ALT, AST, both *p* < 0.05) (Figure 1(a)). Meanwhile, hepatic necrosis was much severe in actively APAP-intoxicated mice than in untreated mice (NAC, MLT, both *p* < 0.05) (Figures 1(b)–1(f)). Additionally, compared with the mice with AILI that received the vehicle, either NAC or MTL could induce a favorable reduction in serum ALT (NAC, MLT, both *p* < 0.05) and AST levels (NAC, MLT, both *p* < 0.05) after AILI (Figure 1(a)). The combination of NAC and MLT resulted in a significant reduction in the levels of serum transaminase (AST, ALT, both *p* < 0.05) and alleviation of liver necrosis (*p* < 0.05), as indicated by both lower necrosis in comparison with NAC monotherapy (Figure 1(g)).

### 3.2. The Add-On Role of MLT Dampens Inflammation Resolution after APAP Overdose

Then, the characteristics of the MLT combined effect on APAP-overdose-induced intoxication were analyzed. The elevated hepatic levels of tumor necrosis factor-*α* (TNF*α*) and IL-6 (both *p* < 0.001) were observed in APAP-overdose mice as well (Figure 1(a)). Accordingly, the single APAP-overdosed mice have a higher level of neutrophil infiltration in the liver. Besides, through flow cytometric analysis, it was found that the volume of hepatic neutrophils was reduced in the combined group after APAP treatment (*p* < 0.01) (Figures 2(b)–2(f)). It appears that a single therapy of NAC or MLT exhibits the same tendency. Nevertheless, there was still no significant difference observed in our data compared with the APAP-induced liver injury group, respectively (*p* > 0.05) (Figure 2(g)).

### 3.3. Treatment of MLT and NAC Attenuates the Decreased GSH Caused by APAP

Given that lipid, the peroxidation in membrane lipids is a typical index for oxidative stress [20]. The next investigation was conducted into lipid peroxidation production. The GSH content characterizes oxidative stress [21]. According to our results, APAP could lead to a sharp decrease of hepatic GSH levels around 6 hours, while the GSH level partially reverses back to normal as time elapsed. It is noteworthy that the addition of MLT to NAC triggers a more effective release in GSH level at 24 hours (*p* < 0.01) (Figure 3(a)). Meanwhile, there are no significant differences in separated treatment groups at an early time points (6 or 12 hours). As indicated by the formation of MDA, APAP is capable of significantly upregulating MDA. As shown in Figure 3(b), APAP-challenged mice manifested a more considerable accumulation in MDA level as time elapsed, compared with the control group (*p* < 0.001), whereas the treatment of adding MLT could enhance the decreased effect of NAC on MDA significantly (*p* < 0.01). Notably, compared with the APAP-challenged group, the add-on of MLT to NAC is more effective in alleviating liver superoxide dismutase (SOD), and catalase (CAT) depletion (all *p* < 0.01) at 24 hours but not in the early time points (Figures 3(c) and 3(d)).

### 3.4. A Combination of the two Reagents Ameliorates APAP-Induced Activation p38/JNK Pathway

An analysis was conducted regarding the effects of MLT addition on NAC-treated liver injury. As shown in Figures 4(a) and 4(b), the level of hepatic phosphate p38 was significantly upregulated in APAP-challenged mice. As expected, the pretreatment with MLT to NAC could also suppress the induction of APAP-treated hepatic RIP1, and JNK phosphorylation is illustrated in Figure 4(a). It can be seen from this figure that the level of phosphorylated JNK was significantly increased in the liver of mice administered with APAP, while there were no significant changes observed in the level of p38 and JNK. Notably, the pretreatment with MLT inhibited the signaling pathway of APAP-evoked hepatic RIP1/JNK.

## 4. Discussion

Due to the absence of the previous experiments on the combination of these two drugs for treating APAP-challenged liver injury. So far, there has been a report that both NAC and MLT can produce a hepatocyte-protective effect on APAP-induced liver injury. As indicated by our data, ALT, AST, and liver necrosis levels were remarkably elevated in these mice. Then a dose of NAC or MLT separately was therapeutically administered, both partially as antioxidant drugs. Since Sener et al. noted that a combination of two drugs plays a beneficial role in hepatic ischemia and reperfusion [22]. Unanimously, it was presented as the damage attenuating role in each medication [6, 17] and manifested a promising liver function recovery when combined with these two reagents in APAP-induced liver injury, suggesting that MLT can enhance the protective effect of NAC. In this study, it found that the add-on of MLT was effective in reversing the APAP-induced liver damage.

Considering that APAP-induced hepatocyte necrosis releases Kupffer cells, monocytes, and neutrophils, the increased level of neutrophils is significant to the hepatic sterile inflammatory response in acute liver injury [23]. Such staining methods could help identify the extent of inflammatory inflammation, which is a limitation of our study. Nevertheless, further evaluation was conducted regarding their effect on hepatic inflammatory infiltration. Though separately applicated, either NAC or MLT has a mild inflammation resolution, it exhibited a promising recovery for neutrophil (Ly6G^+^CD11b^+^) infiltration when adding MLT on NAC. Meanwhile, the combined treatment could also alleviate the release of APAP-induced inflammatory cytokines such as TNF*α* and IL-6. Mechanically, it has been reported that MLT is capable to reverse the tacrolimus-induced increase of TNF*α* and IL-6 [24]. NAC can improve the attraction of TNF*α* and neutrophils in APAP-induced liver injury [9] and inhibit the production of IL-6 in hemodialysis patients [25]. The effect of MLT is mediated through receptor-dependent pathways [26] and regulated by other mechanisms [27]. On the other side, liver cytotoxicity is initiated by the production of NAPQI after APAP-challenge and subsequent generation of proinflammatory cytokines as well as chemokines by Kupffer cells, recruiting neutrophils and monocytes into the liver [9]. Although neutrophils are the first of the liver leukocytes to increase during AILI [28]. it is also thought that neutrophils only have an effect in the early stages and do not contribute to liver injury [29]. Our data support the involvement of neutrophils in the progression of acute liver injury during the early phase of AILI. But our main purpose is to find out the favorable impact of combined drugs in APAP-induced liver injury but not the fundamental mechanism. Thus, the combined therapy method in other hepatic proinflammatory markers and the influx of proinflammatory monocytes remains unknown.

However, the protective effect mediated by melatonin or its metabolites remains inconclusive [30]. MLT and its metabolites all produce the same effect in suppressing ROS [31]. It has a direct antioxidant function or indirectly regulates the anti-oxidative and cytoprotective pathways, despite the rapidly metabolizing in peripheral tissues [32]. Besides, it is also involved in complex anti-oxidative activities by activating NRF2-dependent pathways [33, 34]. In this study, the single dose of melatonin in APAP-related hepatic toxicity failed to recover the hepatic GSH, which is consistent with the previous study [35]. Combined with NAC, however, it reinforces the inhibition in the consumption of GSH, by reportedly elevating *γ*-GCS to increase the intracellular GSH level [16]. The results obtained from this study provide a new therapeutic method for inflammation-related alleviation in liver injury. NAC has a positive effect on the hepatic GSH level exhausted by N-acetyl-p-benzoquinone and reactive oxygen species [1, 2, 36, 37]. MLT plays a limited role in inhibiting GSH depletion [17], which is associated with APAP-induced hepatotoxicity. MLT can induce *γ*-glutamylcysteine synthetase to affect GSH synthesis [16], thus significantly reducing the APAP-induced downregulation of hepatic GSH reductase and GSH peroxidase [17] and displaying an indirect antioxidant function in activating GSH peroxidase [38]. Moreover, this study exhibited a non-pronounced tendency to recovery in single MLT administration, which is confronted with little effect in APAP-related GSH depletion [17].

Concerning the mechanism of APAP-related liver injury, it has been well demonstrated that NAC can partially block the p38/JNK pathway [39]. There is a characteristic activation of JNK involved in APAP-related hepatotoxicity [40]. The RIP1-mediated activation of ASK1-interacting protein 1 (AIP1) is significant to ASK1-JNK/*p*38 apoptotic signaling pathway [41]. RIP1 is upstream of JNK and subsequent cell death [42, 43]. Meanwhile, RIP1 is associated with ROS-induced hepatotoxicity in APAP-related liver injury [44]. MLT is effective in inhibiting the APAP-induced activation of RIP1 and phosphorylation of JNK [17]. APAP could induce the activation of JNK and the phosphorylation of p38 in mouse models [45]. Currently, a conclusion consistent with the previous study is drawn. The overdose of APAP induces an elevation of p38/JNK pathway activation. Despite there being no significant difference observed between these groups for the single use of NAC or MLT, the suppressed APAP-induced phosphorylation of the p38 and JNK, and the combination of two drugs could reverse the activation of p38/JNK pathway, which provides a mechanistic basis for combined therapy.

However, there are also limits to this study. First, there are no clinical species in this study, which will verify the effect of melatonin. Second, the mechanism of this study is not clear, which needs further study to detect it.

## 5. Conclusion

In conclusion, it might produce a more favorable outcome when combined MLT with NAC in APAP-challenged liver injury, thus providing a novel therapeutic method for clinical practice.

## Figures and Tables

**Figure 1:** MLT displays a strengthened role in hepatic protective NAC therapy. (a) Serum level of ALT and AST for each group. H&E staining for wild-type mice (b), single APAP treated mice (c), APAP with NAC treated mice (d), APAP with MLT treated mice (e), and APAP with two drugs (f) and statistical quantification of necrosis in liver tissue for each group (g). The columns are shown as means ± SD (*n* = 6). N represents necrosis area. (^*∗*^*p* < 0.05, ^*∗∗*^*p* < 0.01, ^*∗∗∗*^*p* < 0.001).

**Figure 2:** Enhanced inflammation resolution in mice treated with double drugs. (a) Serum levels of TNF*α* and IL-6 for each group. Representative FACS plots for control wild-type mice (b) (*n* = 6), single APAP treated mice (c), APAP with NAC treated mice (d), APAP with MLT treated mice (e), and APAP with two drugs (f) and statistical quantification of neutrophils in liver tissue for each group (g) (*n* = 5). The columns are shown as means ± SD. (^*∗*^*p* < 0.05, ^*∗∗*^*p* < 0.01, ^*∗∗∗*^*p* < 0.001).

**Figure 3:** The effect of MLT, NAC, and combined treatments on glutathione (GSH) (a), malondialdehyde (MDA) (b), superoxide dismutase (SOD) and (c), catalase (CAT) activities levels (d) at an indicated time. The columns are shown as means ± SD (*n* = 5). (^*∗*^*p* < 0.05, ^*∗∗*^*p* < 0.01, ^*∗∗∗*^*p* < 0.001).

**Figure 4:** The effect of MLT, NAC, and combined drugs in RIP1/JNK associated apoptosis in APAP-induced liver damage. (a) Representative binds and (b) statistical grey-value analysis of protein level for each group. The columns are shown as means ± SD (*n* = 3). (^*∗*^*p* < 0.05, ^*∗∗*^*p* < 0.01).

## Data Availability

The data and materials are available from the corresponding author upon reasonable request.
